This article has been retracted.

# Differential expression of CC chemokines (CCLs) and receptors (CCRs) by human T lymphocytes in response to different *Aggregatibacter actinomycetemcomitans* serotypes

**DOI:** 10.1590/1678-775720150285

**Published:** 2015

**Authors:** Carla ALVAREZ, Alvaro BENÍTEZ, Leticia ROJAS, Myriam PUJOL, Paola CARVAJAL, Jaime DÍAZ-ZÚÑIGA, Rolando VERNAL

**Affiliations:** 1 - Universidad de Chile, Facultad de Odontología, Laboratorio de Biología Periodontal, Santiago, Chile.; 2 - Universidad de Chile, Facultad de Odontología, Departamento de Odontología Conservadora, Santiago, Chile.

**Keywords:** Aggregatibacter actinomycetemcomitans, Chemokines, Chemokine receptors, T-lymphocytes, Th1 cells, Th17 cells

## Abstract

In *Aggregatibacter actinomycetemcomitans*, different serotypes have been described based on LPS antigenicity. Recently, our research group has reported a differential immunogenicity when T lymphocytes were stimulated with these different serotypes. In particular, it was demonstrated that the serotype *b* of *A. actinomycetemcomitans* has a stronger capacity to trigger Th1- and Th17-type cytokine production.

**Objective:**

This study aimed to quantify the expression of different CC chemokines (CCLs) and receptors (CCRs) in T lymphocytes stimulated with the different *A. actinomycetemcomitans* serotypes. In addition, the expression of the transcription factors T-bet, GATA-3, RORC2, and Foxp3, master-switch genes implied in the Th1, Th2, Th17, and T-regulatory differentiation, respectively, was analyzed in order to determine T-cell phenotype-specific patterns of CCL and CCR expression upon *A. actinomycetemcomitans* stimulation.

**Material and Methods:**

Human *naïve* CD4^+^ T lymphocytes were obtained from healthy subjects and stimulated with autologous dendritic cells primed with the different *A. actinomycetemcomitans *serotypes. The expression levels for the chemokines CCL1, CCL2, CCL3, CCL5, CCL11, CCL17, CCL20, CCL21, CCL25, and CCL28, as well as the chemokine receptors CCR1, CCR2, CCR3, CCR4, CCR5, CCR6, CCR7, CCR8, CCR9, and CCR10 were quantified by qPCR. Similarly, the expression levels for the transcription factors T-bet, GATA-3, RORC2, and Foxp3 were quantified and correlated with the CCL and CCR expression levels.

**Results:**

Higher expression levels of CCL2, CCL3, CCL5, CCL20, CCL21, CCL28, CCR1, CCR2, CCR5, CCR6, CCR7, and CCR9 were detected in T lymphocytes stimulated with the serotype *b* of *A. actinomycetemcomitans* compared with the other serotypes. In addition, these higher expression levels of CCLs and CCRs positively correlated with the increased levels of T-bet and RORC2 when T lymphocytes were stimulated with the serotype *b*.

**Conclusion:**

A T-lymphocyte response biased towards a Th1- and Th17-pattern of CCL and CCR expression was detected under stimulation with the serotype *b* of *A. actinomycetemcomitans*.

## INTRODUCTION

In humans, CC chemokines (CCLs) and their specific CC receptors (CCRs) play a central role in physiological and pathological recruitment of immune cells^9^ ^,^ ^24^. During infectious diseases, the expression of CCLs and CCRs produces a chemotactic gradient between regional lymph nodes and infected tissues where, depending on the pattern of CCLs and/or CCRs expressed, specific dendritic cells and T lymphocytes are chemoattracted. Thus, it is established a cellular pathway that goes both ways, in which 1) dendritic cells migrate toward lymphoid organs to present microbial antigens and 2) activated T helper (Th) lymphocytes migrate toward infected tissues to accomplish their specific immunological function^24^.

Th lymphocytes play a central role in the pathogenesis of periodontitis, and a Th1 and Th17-dominated immuno-inflammatory response has been associated with periodontal tissue destruction, alveolar bone resorption, and teeth loss. In this context, the pattern of CCLs and CCRs expressed by Th lymphocytes is crucial in the establishment of the local Th-pattern of immuno-inflammatory response and in the outcome of the disease^9^ ^,^ ^28^. In fact, greater levels of CCL3, CCL4, CCL5, CCL28, CCR1, CCR5, and CCR9 were detected in periodontal lesions of aggressive periodontitis patients, and increased levels of CCL2 and CCR4 were found in lesions of chronic periodontitis patients^8^ ^,^ ^23^. In addition, increased production of IFN-γ has been associated with both greater expression of CCR5 and differentiation of Th1 lymphocytes^16^. Similarly, increased production of IL-6 and IL-23 has been associated with both greater expression of CCL2, CCR6, and CCR7, and subsequent differentiation, migration, and activation of Th17 lymphocytes^13^ ^,^ ^15^. Conversely, increased production of IL-4 and IL-10 has been demonstrated to inhibit the production of CCR5 and to induce the expression of CCL11, CCR3, and CCR4, implied in the Th2 lymphocyte differentiation and function^18^.

Recently, our research group has reported a differential immunogenicity when dendritic cells and T lymphocytes were stimulated with the different serotypes of *A. actinomycetemcomitans* ^2^ ^,^ ^3^. In particular, when T lymphocytes were stimulated with autologous monocyte-derived dendritic cells primed with the serotype *b* of *A. actinomycetemcomitans*, higher levels of Th1- and Th17-associated transcription factors and cytokines were detected compared with similar experiments with the other serotypes, demonstrating that serotype *b* strains of *A. actinomycetemcomitans* have a higher capacity of triggering Th1 and Th17 phenotype and function. It is, therefore, the aim of this investigation to elucidate whether the different serotypes of *A. actinomycetemcomitans* have a role on the differential expression of CCLs and CCRs. We hypothesized that the serotype *b* of *A. actinomycetemcomitans*, when used to stimulate T lymphocytes, induces higher Th1- and Th17-associated CCL and CCR expression when compared with the other *A. actinomycetemcomitans* serotypes.

## MATERIAL AND METHODS

### Experimental design

This experimental study consisted of cell cultures of peripheral *naïve* CD4^+^ T lymphocytes obtained from healthy humans and infected *in vitro* with *A. actinomycetemcomitans*. The protocol of the study was clearly explained to all the participants, who agreed to participate in it by signing an institutional review board-approved informed consent (Protocol 2010/14). The study was conducted in accordance with the Helsinki Declaration of 1975, as revised in 2000.

### *A. actinomycetemcomitans* strains

The *A. actinomycetemcomitans* strains ATCC^®^ 43717™ (serotype *a*), ATCC^®^ 43718™ (serotype *b*), and ATCC^®^ 43719™ (serotype *c*) were cultured on agar brain-heart infusion medium (Oxoid, Hampshire, UK) at 37°C and under capnophilic conditions (8% O_2_ and 12% CO_2_) using an appropriate microaerobic condition generator (CampyGen™; Oxoid, Hampshire, UK). Growth curves were obtained, and live bacteria, having their whole antigenic potentiality, were obtained at the exponential growth phase of the bacterial culture and used for *in vitro *cell stimulation.

### Blood donors

Blood cells were obtained during platelet-apheresis process from healthy donors consecutively enrolled at the Blood Bank of the Hospital Del Salvador in the Eastern Metropolitan Health Service. The study group consisted of 12 adult individuals (seven males and five females, aged 21 to 38 years, mean age of 28.3±5.10 years) who did not have periodontal disease as determined by absence of gingival inflammation, clinical attachment loss, or increased probing depths (PD>3 mm). Further exclusion criteria were the positive test for HIV and hepatitis B or C virus, presence of manifest infections during the last month, fever, symptomatic allergies, abnormal blood cell counts, increased liver enzymes, or medication of any kind except vitamins and oral contraceptives.

### Monocyte-derived dendritic cell generation

For each subject, peripheral blood mononuclear cells (PBMCs) were isolated by density gradient centrifugation using standard procedures (Ficoll-Paque Plus; GE Healthcare, Uppsala, Sweden). For generating a purified population of immature dendritic cells, monocytes were purified from PBMCs by magnetic cell sorting separation (MACS; Miltenyi Biotec, Bergisch Gladbach, Germany). Briefly, PBMCs were incubated with an anti-CD14 monoclonal antibody conjugated to magnetic beads for 15 min at 4°C, loaded onto LS columns and then separated in the magnetic field of a cell separator (MACS; Miltenyi Biotec, Bergisch Gladbach, Germany). The retained CD14^+^ cells, which correspond to monocytes, were then flushed out and washed twice in phosphate-buffered saline. Monocytes were then immediately differentiated to dendritic cells by culturing at 10^6^ cells/mL in RPMI-1640 medium supplemented with 10% foetal calf serum (Gibco Invitrogen Corp., Grand Island, NY, USA) and 20 ng/mL rhGM-CSF and rhIL-4 (R&D Systems Inc., Minneapolis, MN, USA) for 6 d at 37°C.

### T-lymphocyte purification

A purified population of *naïve* CD4^+^ T lymphocytes was obtained from PBMCs by magnetic cell sorting depletion (MACS; Miltenyi Biotec, Bergisch Gladbach, Germany). Briefly, both non-T helper and memory T helper cells were depleted using a cocktail of biotin-conjugated monoclonal antibodies (CD8, CD14, CD15, CD16, CD19, CD25, CD34, CD36, CD45RO, CD56, CD123, TCRγ/δ, HLA-DR, and CD235a) and anti-biotin monoclonal antibodies conjugated to magnetic beads. The magnetically labelled cells were retained within LD columns in the magnetic field of a cell separator (MACS; Miltenyi Biotec, Bergisch Gladbach, Germany), while the unlabelled *naïve* CD4^+^ T lymphocytes ran through.

### Cell stimulation

Monocyte-derived dendritic cells were primed at a multiplicity of infection MOI=10^2^ (bacteria/cells ratio) with different serotypes of *A. actinomycetemcomitans*, and then 10^6 ^T-lymphocytes/mL were activated with primed autologous dendritic cells (50:1) in culture with RPMI-1640 containing 10% foetal calf serum (Gibco Invitrogen Corp., Grand Island, NY, USA) for 5 d at 37°C. Previous to each cell co-culture, dendritic cells were washed twice with RPMI-1640 supplemented with 50 IU/mL penicillin and 50 μg/mL streptomycin (Sigma Chemical Co., St. Louis, MI, USA). T-lymphocyte cultures devoid of dendritic cells or exposed to non-induced autologous dendritic cells were used for comparisons. In each experimental step, dendritic cell and T-lymphocyte counting was performed with a hemocytometer and using a phase contrast microscopy (Axiovert 100; Zeiss Co., Göttingen, Germany), and cell viability equal to or higher than 95% was calculated by Trypan blue dye exclusion. For each individual, the experiment was performed separately.

### Phenotypic cell analysis

T-lymphocyte purification and their subsequent activation were analyzed by flow cytometry (BD FACSCanto™; Becton Dickinson Immunocytometry Systems, San José, CA, USA). Cells were stained using the following monoclonal antibodies conjugated with fluorescein isothiocyanate (FITC) or phycoerythrin (PE): anti-CD4 (CD4^+^ T-lymphocytes), anti-CD25α (activated CD4^+^ T-lymphocytes), anti-CD45RA (*naïve* CD4^+^ T-lymphocytes), and anti-CD45RO (memory CD4^+^ T-lymphocytes) following the manufacturer’s recommendations (BD Biosciences Pharmingen, San José, CA, USA). Isotype-matched control monoclonal antibodies were used to determine the negative cell populations.

### Expression of CD25α, CCR, CCL, and transcription factor mRNAs

From activated T lymphocytes, total cytoplasmic RNA was isolated using 400 µl of ice-cold lysis buffer containing 0.5% Igepal^®^ CA-630 (Sigma-Aldrich, Saint Louis, MO, USA), 50 mM Tris-HCl pH8, 100 mM NaCl, 5 mM MgCl_2_, and 10 mM VRC-40 (Gibco Invitrogen, Carlsbad, CA, USA). Isolated RNA was quantified using a spectrophotometer (Synergy HT; Bio-Tek Instrument Inc., Winooski, VT, USA), and the first-strand cDNA was synthesized using 5 µg of total RNA with a SuperScrip^™^III reverse transcription kit, following the manufacturer’s instructions (Invitrogen, Grand Island, NY, USA). The mRNA expression levels for the chemokines CCL1, CCL2, CCL3, CCL5, CCL11, CCL17, CCL20, CCL21, CCL25, and CCL28, the chemokine receptors CCR1, CCR2, CCR3, CCR4, CCR5, CCR6, CCR7, CCR8, CCR9, and CCR10 and the transcription factors T-bet (Th1), GATA-3 (Th2), RORC2 (Th17), and Foxp3 (T-regulatory), as well as for the activated T-lymphocyte marker CD25α, were quantified by qPCR using the appropriate primers (Figure 1). Briefly, 50 ng of cDNA were amplified using a KAPA^™^ SYBR^®^ Fast qPCR reagent (KAPA Biosystems, Woburn, MA, USA) in a StepOnePlus^®^ equipment (Applied Biosystems, Singapore) as follows: 95°C for 3 min, followed by 40 cycles of 95°C for 3 s, and 60°C for 30 s, and finally a melt curve of 95°C for 15 s, 60°C for 1 min, and 95°C for 15 s, for detection of non-specific product formation and false positive amplification. As an endogenous control, 18S rRNA expression levels were determined.

**Figure 1:** Forward and reverse primers used for CD25α, CCL, CCR, and transcription factor mRNA and 18S rRNA amplifications by qPCR

### Data analysis

The flow cytometry data were analyzed using the WinMDi 2.9 software (The Scripps Research Institute, La Jolla, CA, USA), represented as histograms, and expressed as the percentage of positive cells over the total. The qPCR data were analyzed using the StepOne Software 2.2.2 (Applied Biosystems, Singapore) and presented in fold-change of relative quantities by normalizing the CD25α, CCR, CCL, or transcription factor mRNA expression to 18S rRNA expression using the 2^-ΔΔCt^ method. Data were statistically analyzed using the SPSS 15.0 software (Lead Technologies Inc., Charlotte, NC, USA). The normality of data distribution was determined using the Kolmogorov-Smirnov test. Differences regarding CD expression levels analyzed by flow cytometry were determined using the chi-square test. Differences among groups and within each group regarding the CD25α, CCR, CCL, and transcription factor mRNA expression were analyzed using the Kruskal-Wallis test or ANOVA and Tukey *post-hoc* tests. Correlation coefficients were obtained using the Pearson or Spearman tests. Asterisks were used to graphically indicate statistical significance. A value of p<0.05 was considered statistically significant.

## RESULTS

### T-lymphocyte purification and activation

For this study, highly purified (>98%) populations of *naïve* CD4^+ ^T lymphocytes (CD4^+^CD25α^-^CD45RA^+^CD45RO^-^), devoid of activated or memory CD4^+^ T lymphocytes, were isolated from peripheral blood of healthy donors (Figure 2A). These T lymphocytes activated at a similar extent upon stimulation with dendritic cells primed with the different serotypes of *A. actinomycetemcomitans*, as shown by the similar significant over-expression in CD25α mRNA levels (p<0.001) compared with T lymphocytes exposed to non-induced dendritic cells (Figure 2B). These similar levels of T lymphocyte activation were confirmed at a protein level when the cell-surface expression of CD25α was determined by flow cytometry. In fact, the frequency of CD25α expression (~15%) in T lymphocytes exposed to the different serotypes of *A. actinomycetemcomitans* did not differ significantly (Figure 2C).

**Figure 2:** T-lymphocyte purification and activation. A: T-lymphocyte purification. Flow cytometry analysis of CD4, CD25α, CD45RA, and CD45RO expression demonstrating the purity of *naïve* CD4+ T lymphocytes isolated from healthy donors. B: T-lymphocyte activation. The qPCR analysis for the CD25α mRNA expression in CD4+ T lymphocytes stimulated by autologous dendritic cells primed at a MOI=102 with the *A. actinomycetemcomitans* strains ATCC® 43717™ (serotype a), ATCC® 43718™ (serotype *b*), and ATCC® 43719™ (serotype *c*). C: T-lymphocyte activation. Flow cytometry analysis of the CD25α expression demonstrating the levels of activation of CD4+ T lymphocytes after 5-day stimulation under the same conditions described in Figure 2B. The flow cytometry data from each experiment were expressed as percentage of positive cells over the total, and shown as mean±SD from 4 independent experiments. For relative expression, the CD25α mRNA expression in T lymphocytes cultured in the absence of dendritic cells was considered as 1, as a reference for fold-change in expression. Data are represented as fold-change for 8 independent experiments. Each experiment was performed in duplicate. Comparisons were done *versus* T lymphocytes exposed to non-induced dendritic cells (*p<0.05). *Aa*, *Aggregatibacter actinomycetemcomitans*; CD, cluster of differentiation; DCs, dendritic cells

### Expression of CCLs by *A. actinomycetemcomitans*-induced T lymphocytes

The mRNA expression for the analyzed chemokines was determined by qPCR and represented as fold-change for each condition (Figure 3). When the strain ATCC^®^ 43718™ belonging to the serotype *b* of *A. actinomycetemcomitans* was used for T-lymphocyte activation, higher expression levels of CCL2 (p=0.025 and p=0.024), CCL3 (p=0.003 and p=0.005), CCL5 (p=0.004 and p=0.013), CCL20 (p=0.05 and p=0.02), CCL21 (p=0.001 and p=0.001), and CCL28 (p=0.004 and p=0.008) were detected, when compared with the strains ATCC^®^ 43717™ and ATCC^®^ 43719™ belonging to the serotypes *a* or *c*, respectively. Conversely, when the serotype *a* of *A. actinomycetemcomitans* was used for T-lymphocyte activation, higher expression levels of CCL1 (p=0.008 and p=0.009) and CCL17 (p>0.05 and p>0.05) were detected, when compared with the serotypes *b* or *c*, respectively. CCL11 and CCL25 were not over-expressed in any experimental condition.

**Figure 3:** CC chemokines (CCL) expression by *A. actinomycetemcomitans*-induced T lymphocytes. CCL mRNA expression in T lymphocytes activated by dendritic cells primed at a MOI=102 with the *A. actinomycetemcomitans* strains ATCC® 43717™ (serotype *a*), ATCC® 43718™ (serotype *b*), and ATCC® 43719™ (serotype *c*). For relative expression, the CCL mRNA expression in T lymphocytes exposed to non-induced dendritic cells was considered as 1, as a reference for fold-change in expression (n.i). Data are represented as fold-change for 8 independent experiments. Each experiment was performed in duplicate. Comparisons were done between the different *A. actinomycetemcomitans* serotypes (*p<0.05)

### Expression CCRs by *A. actinomycetemcomitans*-induced T lymphocytes

The mRNA expression for the analyzed chemokine receptors was determined by qPCR and represented as fold-change for each condition (Figure 4). When the serotype *b* of *A. actinomycetemcomitans* was used for T-lymphocyte activation, higher expression levels of CCR1 (p=0.036 and p=0.026), CCR2 (p=0.041 and p=0.042), CCR5 (p=0.029 and p=0.035), CCR6 (p=0.045 and p=0.044), CCR7 (p=0.039 and p=0.020), CCR9 (p=0.040 and p=0.035), and CCR10 (p=0.018 and p=0.022) were detected compared with the serotypes *a* or *c*, respectively. Conversely, when the serotype *a* of *A. actinomycetemcomitans* was used for T-lymphocyte activation, higher expression levels of CCR3 (p=0.006 and p=0.007), CCR4 (p>0.05 and p>0.05), and CCR8 (p>0.05 and p>0.05) were detected, when compared with the serotypes *b* or *c*, respectively.

**Figure 4:** CC receptors (CCR) expression by *A. actinomycetemcomitans*-induced T lymphocytes. CCR mRNA expression in T lymphocytes activated by dendritic cells primed at a MOI=102 with the *A. actinomycetemcomitans* strains ATCC® 43717™ (serotype *a*), ATCC® 43718™ (serotype *b*), and ATCC® 43719™ (serotype *c*). For relative expression, the CCR mRNA expression in T lymphocytes exposed to non-induced dendritic cells was considered as 1, as a reference for fold-change in expression (n.i). Data are represented as fold-change for 8 independent experiments. Each experiment was performed in duplicate. Comparisons were done between the different *A. actinomycetemcomitans* serotypes (*p<0.05)

### Expression of T-bet, GATA-3, RORC2, and Foxp3 by *A. actinomycetemcomitans*-induced T lymphocytes

The mRNA expression for T-bet, GATA-3, RORC2, and Foxp3 was determined by qPCR in T lymphocytes stimulated by dendritic cells primed at a MOI=10^2^ with the different serotypes of *A. actinomycetemcomitans* (Figure 5). Similarly to our previous experiments^2^, T lymphocytes stimulated with the serotype *b* showed a higher relative expression of T-bet (p<0.001 and p<0.001) and RORC2 (p<0.001 and p=0.001) mRNAs than the same cells stimulated with the serotypes *a* or *c*, respectively.

**Figure 5:** Transcription factor expression by *A. actinomycetemcomitans*-induced T lymphocytes. T-bet (Th1), GATA-3 (Th2), RORC2 (Th17), and Foxp3 (T-regulatory) mRNA expression in T lymphocytes stimulated by dendritic cells primed at a MOI=102 with the *A. actinomycetemcomitans* strains ATCC® 43717™ (serotype *a*), ATCC® 43718™ (serotype *b*), and ATCC® 43719™ (serotype *c*). For relative expression, the transcription factor mRNA expression in T lymphocytes exposed to non-induced dendritic cells was considered as 1, as a reference for fold-change in expression (n.i.). Data are represented as fold-change for 8 independent experiments. Each experiment was performed in duplicate. Comparisons were done between the different *A. actinomycetemcomitans* serotypes (*p<0.05)

### Correlation analysis between T-bet, GATA-3, RORC2, and Foxp3 *versus* CCL and CCR expression levels

The correlation analyses between the expression of the transcription factors and the CCLs and CCRs on each activation condition tested (Table 1) yielded positive correlation between T-bet and CCL2, CCL3, CCL5, CCL25, CCR1, CCR2, CCR5, and CCR9, being statistically significant for CCL5 (p=0.049), CCR1 (p=0.040), and CCR2 (p=0.046), when T lymphocytes were stimulated with the serotype *b* of *A. actinomycetemcomitans*. Under the same condition, a positive correlation was also observed between RORC2 and CCL20, CCL21, CCR6, and CCR7, being statistically significant for CCL20 (p=0.041), CCL21 (p=0.004), and CCR7 (p=0.030). In contrast, GATA-3 showed positive correlation with CCL1, CCL17, CCR3, CCR4, and CCR8, being statistically significant for CCL1 (p=0.049), CCL17 (p=0.046), CCR4 (p=0.002), and CCR8 (p=0.048) when T lymphocytes were stimulated with the serotype *a* of *A. actinomycetemcomitans* and with CCR8 (p=0.044) when the same cells were stimulated with the serotype *c*. Foxp3 did not show positive correlation with any CCL or CCR (data not shown). Overall, a T-lymphocyte response biased towards a Th1- and Th17-pattern of CCL and CCR expression was detected under stimulation with the serotype *b* of *A. actinomycetemcomitans*.

**Table 1:** Correlation analysis of transcription factors *versus* CCL and CCR mRNA expressions. The Pearson’s correlation coefficient (r) between the transcription factors T-bet (Th1), GATA-3 (Th2), and RORC2 (Th17) and the Th1-, Th2-, or Th17-associated CCLs and CCRs were calculated using T lymphocytes stimulated by autologous dendritic cells primed at a MOI=102 with the different *A. actinomycetemcomitans* serotypes. *p<0.05

		*Aggregatibacter actinomycetemcomitans*					
		Serotype a		Serotype b		Serotype c	
		r	p-value	r	p-value	r	p-value
T-bet	CCL2	-0.606	0.394	0.918	0.082	-0.487	0.513
	CCL3	-0.755	0.245	0.882	0.118	-0.799	0.201
	CCL5	-0.485	0.515	0.931	0.049*	-0.682	0.318
	CCL25	0.585	0.415	0.909	0.091	0.800	0.200
	CCR1	-0.250	0.750	0.956	0.040*	0.522	0.478
	CCR2	-0.800	0.200	0.934	0.046*	-0.762	0.238
	CCR5	-0.745	0.255	0.882	0.118	-0.966	0.004
	CCR9	-0.971	0.029	0.896	0.104	-0.711	0.289
GATA-3	CCL1	0.920	0.049*	0.837	0.063	0.130	0.870
	CCL11	-0.125	0.825	0.912	0.088	-0.178	0.822
	CCL17	0.934	0.046*	0.519	0.481	-0.072	0.928
	CCL28	-0.231	0.769	0.304	0.696	0.251	0.749
	CCR3	0.880	0.120	0.628	0.372	0.620	0.380
	CCR4	0.998	0.002*	-0.020	0.980	0.578	0.422
	CCR8	0.932	0.048*	0.940	0.060	0.956	0.044*
	CCR10	0.162	0.838	-0.878	0.122	0.144	0.856
RORC2	CCL20	0.897	0.103	0.939	0.041*	0.357	0.643
	CCL21	0.403	0.597	0.996	0.004*	-0.229	0.771
	CCR6	-0.852	0.148	0.875	0.125	-0.717	0.283
	CCR7	0.998	0.002*	0.970	0.030*	0.909	0.091

## DISCUSSION

There is strong evidence suggesting that variations in the host immuno-inflammatory response, in particular, in the T lymphocyte phenotype and function, play an important role in the susceptibility, onset, and severity of periodontitis^6^ ^,^ ^10^. In particular, a Th1 and Th17-dominated immuno-inflammatory response has been associated with the pathogenesis of periodontitis, and an increased expression of Th1- and Th17-related transcription factors and pro-inflammatory mediators have been reported in active periodontal lesions, where alveolar bone resorption is occurring^6^ ^,^ ^17^. In this study, the expression levels of different CCLs and CCRs were analyzed in human *naïve* T lymphocytes, stimulated with dendritic cells primed with different serotypes of *A. actinomycetemcomitans*, demonstrating that the serotype *b* induced greater expression levels of Th1- and Th17-associated CCLs and CCRs, when compared with the other serotypes.

The association between the serotype *b* of *A. actinomycetemcomitans* and the pathogenesis of the periodontitis has been previously analyzed^2^ ^,^ ^3^ ^,^ ^27^ ^,^ ^30^ ^,^ ^32^. In fact, the serotype *b* of *A. actinomycetemcomitans* triggers a greater immunogenic and pathogenic response when in contact with different host cells compared with the other serotypes. For instance, the serotype *b* induces increased resistance to phagocytosis and to killing by macrophages and neutrophils^32^, higher expression of IL-8 and ICAM-1 in gingival epithelial cells^27^, greater production of IL-1β in macrophages^30^, and stronger induction of Th1- and Th17-type of response in dendritic cells and CD4^+^ T lymphocytes^2^ ^,^ ^3^.

To our knowledge, this is the first report associating the different serotypes of *A. actinomycetemcomitans* with a Th1- and Th17-pattern of immuno-inflammatory response by analyzing the CC chemokines and receptors involved in the selective chemo-attraction of Th lymphocytes. These findings are suggestive of the pathogenic role of *A. actinomycetemcomitans* in the aetiology of periodontitis, which may differ among serotypes and specifically let us propose that serotype *b* could play a role in the pathogenesis of the disease by the induction of a local inflammatory environment that favors the specific recruitment of Th1 and Th17 lymphocytes towards the infected periodontal tissues.

In rheumatoid arthritis, which is an inflammatory disease characterized by the development of a Th1 and Th17-dominated immuno-inflammatory response in the affected articular tissues^14^, it has been established that the chronicity of the inflammation is associated with a Th1- and Th17-pattern of CCL and CCR expression. In fact, in chronic inflamed joints, over-expressed levels of CCL2, CCL3, CCL5, CCR1, CCR2, and CCR5, related to a Th1-type response^26^ ^,^ ^29^, and CCL20, CCL21, CCR6, and CCR7, related to a Th17-type response^14^ ^,^ ^22^, have been detected compared with non-inflamed joints. In addition, increased expression of CCL20 has been associated with predominant Th17 lymphocyte infiltration in the affected articular tissues^11^ and, when the chemokine receptors CCR1, CCR2, CCR5, and CCR6 were blocked, a decreased Th1 lymphocyte migration towards the inflamed joints was detected, promoting the resolution of the disease^11^ ^,^ ^26^.

The results of the present study are consistent with the available scientific evidence, and demonstrate that a Th1- and Th17-pattern of immuno-inflammatory response develops during the periodontal infection, at least during an *in vitro* mono-infection with* A. actinomycetemcomitans*. Thus, the Th1 and Th17-dominated immuno-inflammatory response described in periodontitis could be explained by the increased chemo-attraction of recently activated and differentiated Th1 and Th17 lymphocytes from regional lymph nodes and/or by the activation of *naïve* and memory Th1 and Th17 lymphocytes residing in the periodontal tissues^12^ ^,^ ^25^. In this context, the serotype *b* of *A. actinomycetemcomitans* could be associated with local periodontal tissue destruction by the over-production of Th1- and Th17-associated cytokines, such as IL1-β, IL-6, IL-17A, and TNF-α^2^ ^,^ ^3^, and the over-expression of Th1- and Th17-associated CCLs and CCRs, such as CCL2, CCL3, CCL5, CCR1, CCR2, CCR5, and CCR7, as demonstrated in the present study, which are involved in the differentiation and activation of osteoclasts and the resorption of tooth-supporting alveolar bone^6^ ^-^ ^9^ ^,^ ^28^. In fact, a more frequent and higher expression of CCL2 and its specific receptor CCR4 have been reported in chronic periodontitis, and a more prevalent and higher expression of CCL3 and its specific receptor CCR5 have been reported in aggressive periodontitis^9^. Thus, the *A. actinomycetemcomitans* serotype *b*-induced Th1 and/or Th17 lymphocytes could migrate towards infected tissues following the CCL2 and/or CCL3 chemotactic gradient, resulting in a Th1 and/or Th17-associated cytokine production at the periodontal lesion that locally promote the alveolar bone resorption.

The *A. actinomycetemcomitans* strains used in the present study are phenotypically smooth. In fact, these different serotypes correspond to structurally distinct O-polysaccharide components of their respective LPS that function as immuno-dominant antigens. The O-polysaccharide from the LPS produced by the serotype *b* of *A. actinomycetemcomitans* is structurally distinct from the O-polysaccharide produced by the other serotypes. In particular, the O-polysaccharide from serotype *b* consists of a repeating trisaccharide unit composed of α-D-fucose, α-L-rhamnose and β-D-N-acetyl-galactosamine residues, and the O-polysaccharide from serotypes *a* and *c* is composed of 6-deoxy-α-D-talose and 6-deoxy-α-L-talose, respectively^19^ ^,^ ^20^.

Interestingly, our data also show that serotype *b* of *A. actinomycetemcomitans* induces an increment in the CCR10 expression in stimulated T lymphocytes, a chemokine receptor associated with Th2 lymphocyte differentiation and function^31^. In this context, it has been demonstrated that CCR10 is also expressed by Th22 lymphocytes, a recently described T lymphocyte population that complies pro-inflammatory activities^5^; however, this T-cell phenotype has not yet been described in periodontitis. Accordingly, it could be hypothesized that Th22 lymphocytes may be associated with the pathogenesis of periodontitis^1^, which would clarify, at least to a certain degree, the over-expressed levels of CCR10 and its specific chemokine ligand CCL28 detected in the present study. In fact, higher levels of CCL28 have been detected in the gingival crevicular fluid of chronic and aggressive periodontitis patients compared with gingivitis and healthy individuals^4^.

During periodontitis, antigen presentation may occur both in the regional lymph nodes that drain the periodontal tissues and locally in the infected periodontal tissues, in a periodontal site-specific manner. In fact, formation of periodontal lymphoid clusters in which dendritic cells present bacterial antigens to *naïve* or memory T lymphocytes has been reported, promoting the activation and selective differentiation of Th1 and Th17 lymphocytes^12^ ^,^ ^25^. In this scenario, CCR7 and its specific chemokine ligands CCL19 and CCL21 could play a role in the organization of these cellular clusters, as an ectopic lymphoid-like structure^21^, promoting the alveolar bone resorption characteristic of the periodontitis.

## CONCLUSIONS

In T lymphocytes, the serotype *b* of *A. actinomycetemcomitans* induces higher expression levels of chemokines CCL2, CCL3, CCL5, CCL20, CCL21, and CCL28 and of chemokine receptors CCR1, CCR2, CCR5, CCR6, CCR7, and CCR9, when compared with the other serotypes. These increased levels associated with the expression of the transcription factors master-switch genes that trigger the Th1 and Th17 lymphocyte differentiation. Considered together, these data let us propose that variability in the Th1 and Th17 immuno-inflammatory response induced by the different serotypes of *A. actinomycetemcomitans* is associated, at least to a certain degree, with the CC chemokines and receptors that they express; however, functional studies are necessary to confirm our hypothesis.
